# Lightweight forest smoke and fire detection algorithm based on improved YOLOv5

**DOI:** 10.1371/journal.pone.0291359

**Published:** 2023-09-08

**Authors:** Jie Yang, Wenchao Zhu, Ting Sun, Xiaojun Ren, Fang Liu

**Affiliations:** 1 College of Mechanics and Transportation, Southwest Forestry University, Kunming, China; 2 Department of Qingdao Water Group Limited Company, Qingdao, China; 3 College of Economics and Management, Southwest Forestry University, Kunming, China; University of Manitoba, CANADA

## Abstract

Smoke and fire detection technology is a key technology for automatically realizing forest monitoring and forest fire warning. One of the most popular algorithms for object detection tasks is YOLOv5. However, it suffers from some challenges, such as high computational load and limited detection performance. This paper proposes a high-performance lightweight network model for detecting forest smoke and fire based on YOLOv5 to overcome these problems. C3Ghost and Ghost modules are introduced into the Backbone and Neck network to achieve the purpose of reducing network parameters and improving the feature’s expressing performance. Coordinate Attention (CA) module is introduced into the Backbone network to highlight the object’s important information about smoke and fire and to suppress irrelevant background information. In Neck network part, in order to distinguish the importance of different features in feature fusing process, the weight parameter of feature fusion is added which is based on PAN (path aggregation network) structure, which is named PAN-weight. Multiple sets of controlled experiments were conducted to confirm the proposed method’s performance. Compared with YOLOv5s, the proposed method reduced the model size and FLOPs by 44.75% and 47.46% respectively, while increased precision and mAP(mean average precision)@0.5 by 2.53% and 1.16% respectively. The experimental results demonstrated the usefulness and superiority of the proposed method. The core code and dataset required for the experiment are saved in this article at https://github.com/vinchole/zzzccc.git.

## Introduction

Forest is an important part of the Earth’s ecosystem, which can help to maintain the Earth’s ecological balance and promote the development of human society and economy [1]. However, the safety of forest areas has been threatened because of the frequent occurrence of forest fires in recent years. The fires destroyed millions of hectares of forest and devastated the ecological environment, which caused huge economic and animal and plant losses yearly [2]. According to incomplete statistics, there are an average of more than 10,000 forest fires and more than 650,000 hectares of affected forest land in China each year, which caused direct property losses of hundreds of millions of yuan. In 2020, severe wildfires occurred in Australia, which burned at least 19 million hectares, thousands of buildings, and caused the deaths of 34 people and over a billion animals [3]. Forest fires are abrupt strong, destructive, and difficult to tackle usually. Once a fire has broken out, flames can spread freely in the forest area, which is difficult to tackle the fire quickly. If forest fires can be real-time effectively detected and areas of fire smoke can be rapidly identified, it which are helpful for fire-fighters to take measures promptly and control the spread of forest fires. Therefore, how to fastly and accurately detect forest fire and smoke, which is critical for forest fire safety.

Commonly used methods for forest fire prevention include manual patrolling of forest areas and sensor detection. The manual method requires forest rangers to patrol the forest area and find the fire, then report timely it to the relevant departments that take fire extinguishing measures. However, this method has several drawbacks, such as small patrol regions, high-cost consumption, and delayed firefighting, which can result in huge losses. Sensor detection methods for forest fire and smoke detection mainly employ contact fire detectors, such as fire detectors based on chemical sensors [4] and smoke detectors [5], etc. But this method has shortcomings when we detect large-scale forest fires, the detection effect is easily influenced by sensor angles, sensor distances, tree shading, signal transmission, and uncertainties in the surrounding environment. The aforementioned smoke and fire detection techniques are not very effective in providing early warning of forest fires.

With the rapid development of computer vision technology, a large number of video surveillance systems have been installed and employed in forest fire early warning systems. Compared with traditional fire detection technology, video surveillance fire detection technology based on computer vision has the advantages of contactless operation, wide detection range, low maintenance cost, fast response time and good detection performance, etc. The primary goal of this method is to extract the visual features of smoke and fire, such as color [6], texture [7], motion [8], background contrast [9] and the combination of different visual features [10]. However, the fire and smoke detection techniques based on traditional machine learning suffer from many problems, such as complex forest fire images’ background, inconspicuous pixel features, image recognition’s weak generalization and low detection accuracy.

Deep learning techniques in computer vision target detection have made rapid progress since 2012, computers’ computing power increases, especially the Graphics Processing Unit (GPU) rapidly develops, and some excellent public data sets were created and in public use, which brought significant accuracy and efficiency developments and lower computational cost, so deep learning is widely used in the field of smoke and fire detection. These algorithms can be essentially classified into two categories: one is the Two-stage algorithm, whose model structure is divided into two stages. The ROI (region of interest) candidate region is first formed, then the task classification and positioning are performed in this region. Whose classical algorithms include R-CNN [11] (regions with CNN features), Fast-R-CNN [12], and Faster-R-CNN [13]. The other is the One-stage algorithm, which directly predicts the target’s category and position information with a regression-based target detection network. Whose classical algorithms are YOLO (you only look once) series [14] and SSD (single-shot multibox detector) algorithm [15]. In addition, the re-searchers have proposed an improved CNN-based method for smoke and fire detection [16–18]. Recently, researchers start to use Transformer [19] Backbone network to improve neural networks, whose typical ones are ViT (vision transformer) [20], Swin [21] and PVT (pyramid vision transformer) [22]. In the improved process, the pretraining weights from the large-scale image classification database are used as the initial weights for the detector Backbone network, then target detection is performed with Transformer codec-based feature fusion [23, 24]. The Transformer model has good performance, while its computation cost is expensive and it is difficult to train.

The smoke and fire detection technologies based on the above deep learning have achieved good results, but the higher the performance of the detection algorithm, the more convolutional layers of the network structure, the larger the model. In practice, this results in a model with a large number of weighting parameters and low detection efficiency, which is unfavorable for deployment on resource-constrained devices. Therefore, lightweight networks are needed to implement smoke and flame detection. In order to solve the problem of the model’s overlarge and detection efficiency, researchers usually use network pruning [25], knowledge distillation [26], network parameter quantization [27], and the design of lightweight ConvNet. For example, [28] designed a lightweight fire detection network: FireNet, which can run smoothly on low-cost embedded platforms such as the Raspberry Pi. [29] proposed a convolutional neural network based on YOLOv2 for real-time fire and smoke detection in a fire monitoring system, which was deployed in a low-cost embedded device (Jetson Nano) that can be used in a smoke and fire video monitoring system. Furthermore, [30] proposed a deep learning fire recognition algorithm, which was based on model compression and the lightweight network MobileNetV3, which adopted knowledge distillation to improve the accuracy of pruning models, which effectively decreased computational costs in embedded intelligent forest smoke and fire monitoring systems.

Although these lightweight algorithms in the above paper solved the problems of inadequate performance and small applicability in forest smoke and fire monitoring systems, there are still the following problems: (1) If we want to get high detection accuracy in certain cases, then detection methods have a large calculation amount, large model and slow calculation speed, etc. (2) If some lightweight models reduce the number of model parameters, then they are unable to balance accuracy and speed. YOLOv5 is one of the more sophisticated detection algorithms in the YOLO family, which is widely employed in many target identification jobs, it has fast speed, high accuracy and small weight, etc. YOLOv5s has both faster detection speed and higher detection accuracy to meet the requirements of forest fire detection. [31] employed the YOLOv5 detection algorithm for flame detection and optimized the algorithm’s network structure, resulting in effective detection outcomes. However, the large model size and complexity hindered deployment improvements. To address this challenge, this study introduces a lightweight network model based on YOLOv5s for forest smoke and fire detection, with the following main contributions:

- The lightweight C3Ghost and Ghost modules are introduced into the Backbone network and neck network, therefore, the model is compressed while ensuring accuracy and speed of detection.
- The PAN structure is improved by adding learnable weight parameters in feature fusion, which effectively improved the network performance.
- The CA attention mechanism is introduced into the Backbone network to highlight the key information of smoke and fire, at the same time, invalid background information is suppressed, thereby the detection accuracy of the algorithm is improved.

The other main contents of this article are as follows: The second section introduced the YOLOv5 algorithm and improved YOLOv5 algorithm. The third section experiments with the algorithm model before and after improvement. The fourth section discussed the experimental results. The fifth section summarized all the work.

## Method

### YOLOv5s method

The network structure of YOLOv5s is shown in Fig 1. Its structure is mainly di-vided into four parts: image data input, image feature extraction, feature fusion, and image target detection. In the image input stage, the dataset is extended by a series of image enhancement methods such as mosaic and adjusting image brightness. In the image feature extraction stage, the C3 module and the convolution module are used to complete the image extraction operation, and the SPPF module is used to do further dimensionality reduction on the convolutionally extracted information, which can extract higher-order features and enhance the image feature stability. In the feature fusion stage, the PAN (path aggregation network) structure is used to complete the feature fusion of different layers. Finally, three scale detectors are output to detect targets on different scales. The prediction boxes are filtered by NMS (non-maximum suppression), and the highest confidence of prediction box information is retained as the final detection result.

**Fig 1:** YOLOv5s network structure diagram.

### Improvement of YOLOv5s

In order to make the algorithm model run smoothly on resource-constrained embedded devices and improve the speed and accuracy of the smoke and fire, this paper proposes a lightweight fire and smoke detection network based on YOLOv5s. Fig 2 is the improved YOLOv5s structure diagram. The inputs of each module are derived from the outputs of the previous module, and the size of the feature map for each module’s inputs and outputs are unchanged from the unimprovement YOLOv5s. In the Backbone and Neck network, in order to reduce the model size and FLOPs, the ordinary convolution is replaced by the Ghost module [32], and it is embedded in the C3 module to form the C3Ghost module. The CoordAttention [33] (CA) module is embedded after the four C3Ghosts in the Backbone to enhance the feature extraction ability of the network by highlighting the key information of flame detection. In the Neck network, for the purpose of distinguishing the importance of different features in the feature fusion, a number of weight parameters are added in the PAN [34] structure, therefore weight parameters can be learned by the neural network.

**Fig 2:** The structure of the optimized lightweight YOLOv5s model proposed in this paper (added Ghost (①), CA(②), and PAN-weight(③) to the original model).

#### Ghost

Neural network algorithm is difficult to deploy on mobile devices, which has always needed to be solved. The main reason is that the computing ability of mobile devices can-not be compared with that of high-performance GPU devices, which makes it difficult for the existing models to perform the desired performance on mobile devices. While the Ghost module as a new basic unit of the neural network, which can be achieved more feature maps with lower calculation amounts and fewer parameters. The structure is shown in Fig 3.

**Fig 3:** Ordinary convolution and Ghost module.

Fig 3 shows the ordinary convolution method and the Ghost module. There are usually many convolution operations in a convolutional neural network, which leads to large calculation volume, at the same time, the output feature map usually produces redundant features, such as feature map similarity. Suppose the size of the input feature map is h × w × c, then the size of the output feature map is h’ × w’ × n, where h and w represent the height and width of the input feature map respectively, h’ and w’ represent the height and width of the output feature map respectively, and the size of the convolution kernel is k × k. When we use the ordinary convolution method to calculate, the number of FLOPs can be expressed as n × h’ × w’ × c × k × k. When using the Ghost module for computation, a small number of feature maps is generated by the ordinary convolution method, then these generated feature maps need a certain number of cheap transformation operations, finally, the need number of feature maps can be obtained. In the cheap transformation operation, we assume that the channel of the feature map is m (m<<n), the number of transformations is s, and the final number of the obtained new feature map is n. Then we can get Formula (1). Since there is an identity transformation in the transformation process of the Ghost, the actual effective number of transformations is s−1, and Formula (2) can be obtained by eliminating parameter m. It can be known that the FLOPs required for the Ghost are n / s × h’ × w’ × c × k × k + (s– 1) × n / s × h’ × w’ × c × d × d, and d × d is the kernel size in cheap transformation operations. Comparing the Ghost module with the ordinary convolution, we can obtain Formula (3).


n=m×s (1)

$$m\times (s-1)=\frac{n}{s}\times (s-1)$$ (2)

$$\begin{array}{c} r_{s}=\frac{n\cdot h'\cdot w'\cdot c\cdot k\cdot k}{\frac{n}{s}\cdot h'\cdot w'\cdot c\cdot k\cdot k+(s-1)\cdot \frac{n}{s}\cdot h'\cdot w'\cdot d\cdot d}\\ =\frac{c\cdot k\cdot k}{\frac{1}{s}\cdot c\cdot k\cdot k+\frac{s-1}{s}\cdot d\cdot d}\approx \frac{s\cdot c}{s+c-1}\approx s \end{array}$$ (3)

Obviously, the FLOPs number of the ordinary convolution is s times that of the Ghost module from Formula (3). So we can apply the Ghost module to replace the ordinary convolution to achieve the purpose of lightweight in the detection network. The structure for inserting the Ghost is shown in Fig 4. Fig 4(A) is the structure of the unchanged algorithm C3 module, and different BottleNeck can constitute different C3 structures. When the BottleNeck is replaced by GhostBottleNeck to form the C3Ghost structure (Fig 4(B)), while other ordinary convolutions are replaced by the Ghost module in the network, then we can realize compressing the size of the model and reducing the amount of calculation.

**Fig 4:** C3 module and C3Ghost.

#### Coordinate attention

The essence of the attention mechanism is highlighting the importance of the detection target and suppressing irrelevant background region information by increasing the weight of the model’s interest region. CA is a novel, lightweight, and efficient attention mechanism module, which is used to improve the performance of the model, and can be more easily embedded in the network model, with virtually no additional computational effort. The structure is shown in Fig 5.

**Fig 5:** The structure of coordinate attention.

The CA module is divided into two steps: coordinate information embedding and coordinate attention generation. Firstly, each channel is encoded respectively from horizontal and vertical directions through X_Avg Pool and Y_Avg Pool operations (Formula (4)(5)). Where *z*_*c*_^*h*^*(h)* and *z*_*c*_^*w*^*(w)* respectively represent the outputs of the *c*th channel’s *h* height and *w* width, and *x*_*c*_ represents the input.


$$z_{c}^{h}(h)=\frac{1}{w}\sum_{0\leq i\leq w}x_{c}(h,i)$$ (4)

$$z_{c}^{w}(w)=\frac{1}{h}\sum_{0\leq i\leq h}x_{c}(j,w)$$ (5)

Secondly, connecting the feature maps generated from the first step, then the connected feature maps are transformed by using a 1 × 1 convolutional transform function F_1_ (Formula 6). Where *δ* is a nonlinear activation function, and *f* is an intermediate feature map that encodes spatial information in the horizontal and vertical directions. The *f* is sliced to two separate tensors (*f*^*h*^ ∈ *R*^*c/r*×*h*^ and *f*^*w*^ ∈ *R*^*c/r*×*w*^) from two dimensions, then the feature maps *f* ^*h*^ and *f* ^*w*^ are transformed into original channel number *c* with a 1 × 1 convolutional transformation functions *F*_*h*_ and *F*_*w*_, calculating as in Formula (7)(8). *σ* in the formula represents the sigmoid activation function. In addition, *r* is used to reduce *f* ‘s channel number to reduce the model’s complexity and calculation consumption.


$$f=\delta (F_{1}([z^{h},z^{w}]))$$ (6)

$$g^{h}=\sigma (F_{h}(f^{h}))$$ (7)

$$g^{w}=\sigma (F_{{}^{w}}(f^{w}))$$ (8)

Finally, *g*^*h*^ and *g*^*w*^ outputs are extended as the outputs of different attention weights, then Coordinate Attention Block can be written as:

$$y_{c}(i,j)=x_{c}(i,j)\times g_{c}^{h}(i)\times g_{c}^{w}(j)$$ (9)

#### PAN-weight

YOLOv5 completes the different scales’ feature fusion with PAN method. Usually, which only is a simple feature maps’ ‘concat’ operation during the feature fusion process, while the importance of the added feature maps isn’t differentiated. The input feature maps are from different convolutional layers during the feature fusion, which brings about different contributions to the output feature map, therefore a simple feature maps’ ‘concat’ operation maybe not the best way here.

This paper proposes a simple and efficient weighted feature fusion mechanism. A weight parameter is added to each input, which can be learned by the neural network to distinguish the importance of different features during feature fusion (Fig 6). Whose calculation is shown in Formula (10) (11) (Taking *P*_*2*_^*td*^ and *P*_*2*_ for example). Where *C* and *P* respectively represent the input and output features of the current layer, and *P*^*td*^ represents the intermediate features, and *w* represents the weight parameter learned by the network, and the *Resize* operation represents up-sampling or down-sampling, and *ε* is a small value to avoid numerical instability.


$$P_{2}{}^{td}=Conv(\frac{w_{1}\cdot C_{2}+w_{2}\cdot Resize(C_{3})}{w_{1}+w_{2}+\varepsilon })$$ (10)

$$P_{2}=Conv(\frac{w\prime_{1}\cdot P_{2}{}^{td}+w\prime_{2}\cdot Resize(P_{1})}{w\prime_{1}+w\prime_{2}+\varepsilon })$$ (11)

**Fig 6:** PAN-weight.

## Math

### Experiments introduction

Model training and model testing of this paper’s experiments are conducted on Ubuntu 20.04 operating system. The GPU of the device is GeForce RTX2060 12G, and the CPU is i5-12490F, and the RAM is 16G. The software environment is pytorch 1.8.1, CUDA 10.2, cudnn 7.6.5 and python 3.8.

All input images’ size in the experiments is 640 × 640 × 3. In the part of image enhancement, the adopted methods are recommended from the original algorithm, such as mosaic, and adjusting HSV parameters, which are used to expand and diversify the input training network images.

Warmup training is used for all experimental learning rate. The specific method is to rapidly increase the learning rate from 0 to 0.01 in the early training stage’s 0 to 3 epochs. In order to avoid the model’s oscillation problem at the beginning of the training phase that can make it difficult to converge, a large learning rate in the early stage is required. SGD (stochastic gradient descent) is used as an optimizer to update and optimize the model’s weight. The specific parameters are set as follows: batch size to 128, initial learning rate to 0.01, momentum parameter to 0.937, weight attenuation factor to 0.0005, and 500 training epochs.

The common evaluation metrics in target detection tasks are precision and recall. Precision indicates the predicted targets’ proportion of the correct to all in the forecast targets. Recall indicates the correct target’s proportion of the predicted to all in the fore-cast targets. The calculation formulas are as follows:

$$precision=\frac{TP}{TP+FP}$$ (12)

$$recall=\frac{TP}{TP+FN}$$ (13)

where *TP*, *FP*, and *FN* respectively denote true positive, false positive, and false negative. mAP is a measurement indicator combining precision and recall, which is adopted in this experiment, whose value ranges from 0 to 1. The calculation method is as follows:

$$\text{mAP}=\frac{1}{C}\sum_{k=1}^{N}P(k)\Delta R(k)$$ (14)

where *N* denotes the number of samples in the test set, and *P* denotes precision, and k denotes the k sample, and *△R(k)* denotes the change in recall *R* from the *k-1* sample to the *k* sample, and *C* denotes the classes’ number to be identified in the multiclassification detection task.

We set IoU = 0.6 to evaluate the model’s performance metrics such as precision, recall, and mAP. The Parameter size and inference time per image are also used to evaluate the weight and speed of the model.

### Experimental results on the dataset

The number of datasets adopted in this experiment was 11,667, which were randomly divided into training, validation, and test set, whose number respectively was 8,494, 2,114, and 1,059. There were two main dataset sources: (1) video and images dataset captured from the web, (2) self-collected tree burning dataset. The web-captured and self-collected videos were first processed by frame extraction (30 frames apart), and the video extracted by frame was added to the image dataset, and the image dataset was labeled with LabelImg tool, then the final dataset for this experiment was formed. The scene mainly includes forest fires of daytime, dusk, and nighttime in the image dataset. Some of the image data is shown in Fig 7.

**Fig 7:** Partial dataset display.

The instances of the experimental dataset are labeled into ’smoke’ and ’fire’ (Table 1) categories, where ’smoke’ easily spread, resulting in a relatively small percentage of its population. The experiments employ a larger dataset and classification instances, which can avoid the detrimental effects when ‘smoke’ and ‘fire’ sample numbers are unbalanced, at the same time, which can fully extract the features of each classification.

**Table 1:** Number of dataset instances.

labels	instances
smoke	8693
fire	16232

Multiple sets of control experiments were conducted to find the optimal network structure and to test changes in performance caused by changes in the network structure. in order to find the Ghost module’s optimal embedding position and to highlight the effect of PAN-weight on model performance, five controlled groups experiments were conducted, which were: YOLOv5s, YOLOv5s_Ghost_all, YOLOv5s_Ghost_backbone, YOLOv5s_neck and YOLOv5s_Ghost_all_PAN-w. The results are respectively shown in Fig 8 and Table 2.

**Fig 8:** Experimental results of each model.

**Table 2:** The result of different models.

Model	Precision	Recall	mAP@.5	mAP@.5:.95	FLOPs(G)	Speed (ms)	Weight(M)
YOLOv5s	0.87	0.827	0.863	0.559	15.8	3	14.3
YOLOv5s_Ghost_backbone	0.876	0.819	0.865	0.553	10.6	2.7	10.5
YOLOv5s_Ghost_neck	0.885	0.817	0.864	0.573	13.2	2.9	11.6
YOLOv5s_Ghost_all	0.882	0.811	0.86	0.559	8	2.7	7.7
**YOLOv5s_Ghost_all_PAN-w**	**0.889**	**0.81**	**0.868**	**0.565**	**8.2**	**2.7**	**7.9**

Fig 8 shows the training process of different models on the dataset, and Table 2 shows the performance of the models on the test set. The Ghost module has a small variation of Precision, Recall, mAP@0.5, and mAP@0.5:0.95 metrics within 1.6% at different embedding locations. The lightweight of YOLOv5s_Ghost_all model becomes more outstanding when it is embedded with more Ghost modules. Compared with YOLOv5s, the FLOPs and weight parameters are respectively reduced by 49.36% and 46.15%, and the running speed increases by 10%. In addition, YOLOv5s_Ghost_all_PAN-w adds a PAN-weight structure to YOLOv5s_Ghost_all, which makes model performance significant improving. It can be concluded that the YOLOv5s_Ghost_all_PAN-w network model has better model performance and lightness.

Four groups of control experiments were set to find the best embedding position of the CA modules. The CA modules were respectively embedded in the Backbone (behind each C3Ghost module: CA_Backbone_①, and behind the last C3Ghost module: CA_ Backbone_②), Neck (behind each C3Ghost module: CA_Neck), and all (behind each C3Ghost module in the whole network: CA_All) of the YOLOv5s_Ghost_all_PAN-w model. Table 3 shows the results of these four experiments. According to the result, the first group of experiments is better and has a certain improvement in the performance of the network model. It can be concluded that the model can obtain the best detection performance when the CA module is added behind each C3Ghost in the Backbone network.

**Table 3:** Comparison results of the CA module in different positions.

Model	Precision	Recall	mAP@.5	mAP@.5:.95	FLOPs(G)	Speed (ms)	Weight(M)
**CA_Backbone_①**	**0.892**	**0.827**	**0.873**	**0.566**	**8.3**	**2.7**	**7.9**
CA_ Backbone_②	0.887	0.811	0.865	0.558	8.3	2.5	7.8
CA_Neck	0.884	0.825	0.862	0.561	8.3	2.7	7.9
CA_All	0.889	0.816	0.863	0.562	8.4	2.8	8

Fig 9 shows the performance comparison of the proposed method and YOLOv5s in different scenarios. Grad-CAM [35] helps to visually interpret the trained model, and it can observe which region of the network more is focused on. From Fig 9, smoke and fire detection in the forest can be well achieved by YOLOv5s and our proposed method, in the meantime, more attention to the model and the corresponding confidence can be obtained with our proposed method. The results show that our proposed method is superior to YOLOv5s.

**Fig 9:** Comparison of YOLOv5s and our method detection results.

### The comparison results with related methods

In order to further validate the performance of proposed method in this paper, we compare it with the commonly used classic lightweight network YOLOv3-tiny and YOLOv5n. Meanwhile, we compare it with other YOLOv5s lightweight schemes (MobileNetv3-small [36], Shufflev2 [37], etc. are added to YOLOv5s as a Backbone, and the obtained new models are respectively named YOLOv5s-M and YOLOv5s-S here). The results are shown in Table 4.

**Table 4:** Compare with other lightweight networks.

Model	Precision	Recall	mAP@.5	mAP@.5:.95	FLOPs(G)	Speed (ms)	Weight(M)
YOLOv3-tiny	0.834	0.762	0.814	0.437	12.9	1.9	17.4
YOLOv5n	0.812	0.79	0.823	0.475	4.1	1.5	3.8
YOLOv5s-M	0.778	0.688	0.762	0.4	2.3	1.8	3.1
YOLOv5s-S	0.774	0.72	0.759	0.387	1.8	1.2	1.9
YOLOv5s	0.87	0.827	0.863	0.559	15.8	3	14.3
**Ours**	**0.892**	**0.827**	**0.873**	**0.566**	**8.3**	**2.7**	**7.9**

It can be seen from Table 4, comparing with other lightweight methods, the proposed method in this paper obtains better performance when a faster running speed is ensured. Comparing with YOLOv5s, the proposed method can respectively reduce model size and FLOPs by 44.75% and 47.46%, while precision and mAP@0.5 respectively increase by 2.53% and 1.16%. YOLOv3-tiny achieves faster running speed, while it has a poorer performance in model size and precision. And YOLOv5n, YOLOv5s-M, and YOLOv5s-S have greater lightweight advantages, but their precisions respectively are only 91.03%, 87.21%, and 86.77% of the proposed method in this paper. It can be concluded that the method proposed in this paper has more significant advantages than other lightweight networks.

In addition to the CA attention mechanism, other attention mechanisms were adopted in this experiment, such as CBAM (Convolutional Block Attention Module) [38], ECA (Efficient Channel Attention) [39], and SE (Squeeze-and-excitation) [40]. The experimental results are shown in Table 5. Obviously, the CA module can more improve the network model’s performance than other attention mechanisms.

**Table 5:** Compare with other lightweight networks.

Model	Precision	Recall	mAP@.5	mAP@.5:.95	FLOPs(G)	Speed (ms)	Weight(M)
+CBAM	0.882	0.816	0.87	0.569	8.3	2.8	8
+ECA	0.888	0.813	0.864	0.566	8.3	2.5	7.9
+SE	0.888	0.812	0.863	0.561	8.3	2.5	8
**+CA (ours)**	**0.892**	**0.827**	**0.873**	**0.566**	**8.3**	**2.7**	**7.9**

## Discussion

Tables 2 and 3 show the influence of the proposed improved method on the whole algorithm performance through ablation experiments. YOLOv5s_Ghost_backbone denotes that the C3Ghost and the Ghost modules are only introduced into the Backbone network. YOLOv5s_Ghost_neck denotes that the C3Ghost and the Ghost modules are only introduced into the neck network. These two models not only contribute to reducing the model’s parameters and improving the network performance, but the introduced number of the Ghost modules is fewer, and the model’s lightweight limits. YOLOv5s_Ghost_all denotes that the C3Ghost and the Ghost modules are introduced into the whole network. The experimental results show that the improved network model has a significant improvement in lightweight. Whose main reason is that the Ghost module replaced the ordinary convolution, which can greatly reduce the parameters’ number to be computed in the network, meanwhile, the performance of feature extraction and feature understanding become better. YOLOv5s_Ghost_all_PAN-weight represents an improvement on YOLOv5s_Ghost_all with PAN-weight, where features in different layers are set with a learnable weight parameter during the fusion process, thus the network performance significantly improves. In addition, this paper experiments with the embedding position of the CA modules. Ac-cording to the experimental comparison, we can get better detection performance when the CA module is embedded behind C3Ghost module of Backbone, which can highlight the target’s detection information and suppress other useless information in feature extraction phase. Fig 9 shows that both the proposed method and YOLOv5s can achieve better smoke and fire detection in the forest, but the proposed method has better detection performance from the obtained corresponding confidence.

Table 4 shows the comparison results of the proposed method in this paper with other lightweight methods. YOLOv3_tiny uses methods of image preprocessing, feature extraction, and feature fusion, but its performance lags behind the proposed method in YOLOv5, resulting in a poorer effect. Although YOLOv5n, YOLOv5s-M and YOLOv5s-S have more outstanding lightweight performance, their fewer parameters lead to insufficient feature extraction performance in the Backbone network, which brings unsatisfactory detection performance. Table 5 shows that the CA module provides the greatest performance improvement for the proposed network model, comparing to other attention mechanism modules.

## Conclusions

In this paper, a lightweight forest smoke and fire detection model based on YOLOv5s is proposed. The main conclusions are as follows.

- The C3Ghost and the C3 module were introduced into the YOLOv5s network, which maintained the network’s detection performance and effectively reduced the number of model parameters.
- The PAN structure in YOLOv5s network was improved by adding learnable weight parameters in feature fusion, which effectively improved the network performance.
- The CA attention mechanism was employed in the network feature extraction process, which effectively improved the model’s detection accuracy.
- Comparing with other lightweight methods and other attention mechanisms, the proposed method had better detection performance for smoke and fire in the forest.

The experimental results show that the proposed method has a lightweight structure, higher accuracy, and can satisfy real-time requirements. At the same time, the lower computational cost makes the model easy to deploy to resource-constrained devices for smoke and fire detection in large area’s forests, which has positive significance for timely detecting fire sources and preventing large-area fires.

In our future work, we will consider further improving the algorithm by introducing more advanced technologies and ideas to enhance detection performance and accuracy. We can also explore how to effectively detect smoke and fires in different environments and lighting conditions. Additionally, we can further optimize the computational efficiency and speed of the algorithm to meet the demands of practical application scenarios.
